# Clinical Manifestations of Ultrasonic Virtual Reality in the Diagnosis and Treatment of Cardiovascular Diseases

**DOI:** 10.1155/2021/1746945

**Published:** 2021-06-25

**Authors:** Hairong Chen, Qiuguo Zou, Qi Wang

**Affiliations:** ^1^Department of General Practice Medicine, Affiliated Haikou Hospital of Xiangya Medical College of Central South University, Haikou, Hainan 570208, China; ^2^Department of Ultrasonic Medicine, Affiliated Haikou Hospital of Xiangya Medical College of Central South University, Haikou, Hainan 570208, China

## Abstract

On a global scale, cardiovascular disease has become one of the most serious diseases that endangers human health and causes death and seriously threatens human life and health. If we can make accurate, timely, and effective judgments on cardiovascular-related parameters and take corresponding effective measures, the incidence of cardiovascular diseases can be reduced to a large extent. Based on this, this paper proposes the clinical application research of ultrasound virtual reality technology in the diagnosis and treatment of cardiovascular diseases. This article uses literature methods, experimental research methods, mathematical statistical analysis methods, and other research methods and in-depth study of virtual reality technology, cardiovascular disease, and other theoretical knowledge and briefly introduces ultrasound image denoising algorithms, such as bilateral filtering and PM model. And on this basis, it establishes clinical trials of ultrasound virtual reality technology in the diagnosis and treatment of cardiovascular diseases. This article mainly analyzes the application of virtual reality technology, technology comparison, and the experimental results carried out in this article. From the survey results, the total prevalence of hypertension was 25.1%, and the prevalence of males and females was 25.9% and 24.4%, respectively; the diagnostic accuracy rate of the experimental group reached 85.39%, while the diagnostic accuracy rate of the control group was 76.8%. It shows that the use of ultrasound virtual reality technology for disease diagnosis can effectively improve the accuracy of cardiovascular disease diagnosis and reduce the proportion of misdiagnosis and missed detection.

## 1. Introduction

Cardiovascular disease has become the number one killer of Chinese people's health. In recent years, China has been in a period of rapid social and economic development. With the acceleration of social changes and the gradual acceleration of population aging, people's living standards and behavior patterns have undergone tremendous changes. Bad habits such as insufficient exercise, drinking, smoking, and improper eating habits have caused many diseases. For example, cardiovascular disease is one of the most morbidity types, which seriously endanger people's health and lives.

The development of virtual reality and augmented reality technology is an innovative development for all walks of life. In medicine, full use of virtual reality technology, for interns, can adjust according to their own needs and perform simulated surgery to increase clinical experience. The creation of a good virtual medical environment provides a brand-new experience for patients and provides more opportunities and possibilities for patients' treatment.

The age of onset of Huo X type 2 diabetes is declining. Since non-Chinese patients with early-stage type 2 diabetes (defined as <40 years of age) have an increased risk of vascular complications, they investigated the impact of early-stage type 2 diabetes on the risk of nonfatal cardiovascular disease. They conducted a cross-sectional survey using data from China's National HbA1c Surveillance System (CNHSS), including 222 to 773 Chinese type 2 diabetes patients from 630 hospitals in 106 cities in 30 provinces in China in 2012. They recorded demographic information and clinical data. Nonfatal cardiovascular disease is defined as nonfatal coronary heart disease or nonfatal stroke. The prevalence of nonfatal cardiovascular diseases was standardized for the Chinese population in 2011. They performed logistic regression analysis to obtain the odds ratio (OR) of cardiovascular disease risk in patients with early-onset and late-onset type 2 diabetes. Because CNHSS does not include patients who only receive diet or lifestyle therapy, it does not capture information about smoking or blood lipids. Therefore, their experiment is not of great practical use for the treatment of diabetic patients, and a larger experimental basis is needed [1, 2]. Maples-Keller JL learning goal: after participating in this activity, learners should be able to better evaluate the literature on the effectiveness of incorporating virtual reality (VR) in the treatment of mental illnesses, evaluate the use of exposure-based interventions for anxiety disorders, and evaluate virtual reality (VR) enables users to experience a sense of presence in a computer-generated three-dimensional environment. Sensory information is transmitted through head-mounted displays and dedicated interface devices. These devices track the movement of the head in order to change the movement and the image in a natural way with the movement of the head, thereby making people feel immersed. VR allows the therapist to control the delivery of sensory stimuli and is a convenient and cost-effective treatment method. This review focuses on the existing literature on the effectiveness of including VR in the treatment of various psychiatric disorders, with a particular focus on exposure-based interventions based on anxiety disorders. A systematic literature search was conducted to identify the research being carried out. The research is very innovative, but there is still a lack of effectiveness in the treatment of mental illness [3, 4]. Dale J explores the use of musculoskeletal ultrasound (MSUS) to assess disease activity to improve the strategy of intensive targeted therapy (T2T) for early rheumatoid arthritis (RA). A new diagnosis of RA or undifferentiated arthritis (symptom duration <1 year) was randomly assigned to aim to achieve DAS28-erythrocyte sedimentation rate (ESR) < 3.2 (control) in the combined DAS28-ESR/MSUS assessment (intervention) or the total power Doppler joint, the strategy of the total count ≤ 1. If the following conditions are met, it means that the MUS examination has been performed: DAS28-ESR < 3.2 or DAS28-ESR ≥ 3.2, and two joints are swollen. Gradually standardize and take anti-rheumatic drugs (DMARD), such as methotrexate monotherapy, triple therapy, and etanercept/triple therapy, to improve the condition. The core set variables of the American College of Rheumatology (ACR) are evaluated 3 times a month by meteorologists who are unaware of the group assignment. MRI scans of the main hands and wrists were performed at baseline and at 18 months, and radiographs of the hands and feet were taken. Two readers used the outcome indicators in rhubarb for grading. Although his research mainly uses musculoskeletal ultrasound facilities, he has not implemented ultrasound research, and the research remains to be insufficient [5].

The innovations of this article are (1) combining theory with practice, fully applying theoretical foundations in practice, and discussing the application of virtual reality technology to the diagnosis and treatment of cardiovascular diseases; (2) qualitative and quantitative research combined, there are both data analysis and qualitative content analysis.

## 2. The Clinical Application Method of Ultrasound Virtual Reality Technology in the Diagnosis and Treatment of Cardiovascular Diseases

### 2.1. Cardiovascular Disease

Cardiovascular disease, well known as a circulatory system disease, is a series of diseases including the circulatory system. The circulatory system refers to the organs and tissues that transport blood to the human body, mainly including the heart and blood vessels (arteries, veins, capillaries, etc., which are divided into acute and chronic, usually related to arteriosclerosis) [6]. The current diagnosis mainly relies on some inspection items, which are judged by doctors based on experience. However, because cardiovascular diseases are related to all parts of the body, only the usual cardiac examinations include electrocardiogram, dynamic electrocardiogram, chest X-ray, and heart color Doppler ultrasound, in addition to myocardial enzymes, myocardial antibodies, coronary angiography, exercise treadmill test, coronary CT, myocardial radionuclide imaging, and myocardial biopsy [7]. Therefore, in practice diagnosis and treatment, taking into account the cost and time and other issues, not all examinations must be carried out, usually by the doctor based on experience to select some of them [8]. Moreover, usually, the outpatient doctors focus on a certain special field, and it is inevitable that they have their own blind spots for system-level diseases such as cardiovascular disease. Therefore, missing some important inspection items may lead to diagnostic errors [9].

In addition, any disease is the result of environmental factors and genetic factors, and cardiovascular disease is no exception. Interheart studies a total of 29,000 patients in 52 countries around the world. According to the results of the study, 90% of cardiovascular diseases are related to environmental factors, and genetic factors account for only 10% [10, 11]. High cholesterol, smoking, diabetes, high blood pressure, abdominal obesity, insufficient exercise, insufficient fruits and vegetables in the diet, mental stress, and heavy drinking are currently known risk factors that can be changed. These risk factors can predict 90% of the risk of myocardial infarction. By controlling these risk factors, the risk of myocardial infarction can be reduced by 80%. Moreover, in treatment, different treatment methods can be adopted for different individual causes [12]. Therefore, etiological assessment is an effective method to identify high-risk groups. Etiological intervention can effectively reduce the morbidity and health risks of high-risk groups, thereby delaying the occurrence of diseases [13, 14]. However, with the current way of doctors looking, smelling, asking, and cutting, it is easy to ignore some risk factors and affect the prevention and treatment effects [15].

Cardiovascular function parameters are an important way to detect cardiovascular diseases. The detection is relatively accurate, but the risk is high, so it is only suitable for severely ill people and cannot be widely used in medical treatment [16, 17]. There are many methods to detect cardiovascular function clinically, including CT scan examination, electrocardiogram detection, echocardiography, and nuclear magnetic resonance; these methods can effectively detect cardiovascular function to effectively control cardiovascular disease, but these detection instruments are not only cumbersome to operate but also costly and are not suitable for general household use. Therefore, the study of simple and economical diagnostic methods and devices for cardiovascular function is very important for the effective prevention and control of cardiovascular diseases [18, 19].

### 2.2. Ultrasound Technology

#### 2.2.1. Brief Description of Ultrasound Technology

The changes in people's diet and living habits in modern society have led to the occurrence of cardiovascular system diseases. These diseases are not easy to be detected in the initial stage of onset, which makes cardiovascular system diseases have a higher mortality rate [20]. Generally speaking, sound is the result of a kind of mechanical wave propagating in the air to human ears. This mechanical wave may cause the tympanic membrane to vibrate [21]. Under normal circumstances, the dynamic wave of the vibration frequency of the human eardrum must be 20 Hz to 20 kHz. Ultrasonic waves refer to mechanical waves whose mechanical frequency exceeds 20 kHz. Ultrasound used in medicine usually selects 2.5–13 MHz as the main frequency application range [22].

Ultrasound is a kind of mechanical wave. The main application types of ultrasonic are Lamb wave, surface wave, transverse wave, and longitudinal wave. Since transverse waves cannot propagate in air and liquids, under normal circumstances, high-frequency ultrasound has good directional propagation characteristics [23, 24]. At the same time, ultrasonic waves have the characteristics of propagating and reflecting sound waves. When ultrasonic waves pass through the two-way interface at a vertical angle, part of the ultrasonic waves may enter the second medium through the interface [25, 26]. The propagation continues to become a propagating wave, and the propagation direction of the ultrasonic wave does not change. The other part of the ultrasonic wave propagates and reflects in the opposite direction to the adjacent wave on the interface and becomes a reflected wave [27, 28]. Due to the nature of ultrasound, ultrasound detection is possible. Medical ultrasound diagnosis is also divided into transmission method and reflection (echo) method according to the propagation mode of ultrasound.

Ultrasonic echo tracking technology uses the propagation characteristics of ultrasound in the human body to sample the ultrasound echo signal and perform relevant filtering on the sampled signal. [29]. This technique utilizes the convenient and nondestructive advantages of ultrasound and has very important application value in the detection of blood vessel elasticity.

#### 2.2.2. Ultrasound Image Denoising Algorithm

*(1) Elastic Signal-to-Noise Ratio (SNRe) and Elastic Image Contrast-to-Noise Ratio (CNRe)*. A large number of experiments have proved that the elastic signal-to-noise ratio (Signal-to-Noise Ratio elastography, SNRe) and the elastic image contrast-to-noise ratio (Contrast-to-Noise Ratio elastography, CNRe) are effective and important two for evaluating the quality of ultrasound images. SNRe is the ratio of the mean value to the standard deviation of a uniform area in the image, and it usually reflects the ratio of image signal to noise intensity. CNRe is used to indicate the ability to detect the lesion area. This parameter is often used clinically to distinguish the normal tissue area of the human body from the diseased tissue area, reflecting the degree of easy identification of the two areas [30]. The mathematical expressions of SNRe and CNRe are as follows:

(1) $$\begin{array}{c} \text{SNRe}=\frac{\varpi }{\vartheta },\\ \text{CNRe}=\frac{\left[2\left(\varpi_{a}-\varpi_{b}\right)\right]}{\left(\vartheta_{a}^{2}+\vartheta_{b}^{2}\right)}. \end{array}$$

In the formula, *ϖ* and *ϑ*, respectively, represent the image mean and standard deviation; the following tables *a* and *b*, respectively, point to the characteristic area and the background tissue area. *ϖ*_*a*_ and *ϑ*_*a*_, respectively, represent the mean value and standard deviation of the image feature area (i.e., lesion area); *ϖ*_*b*_ and *ϑ*_*b*_, respectively, represent the mean value and standard deviation of the background area (i.e., noise area) consistent with the size of the feature area.

The elastic signal-to-noise ratio growth rate (SNRe′) and the elastic image contrast-to-noise ratio growth rate (CNRe′) refer to the growth rate of the image quality measurement. The larger the value, the faster the image quality growth. SNRe′ is to calculate the SNRe value of the original image and the denoised image according to the expression and then obtain the change value of the elastic signal-to-noise ratio before and after the image is denoised; in the same way, CNRe′ is the CNRe of the original image and the denoised image. The value is calculated according to the expression, and then the change value of the contrast-to-noise ratio of the elastic image before and after the image denoising is obtained. Its definition expression is as follows:

(2) $$\begin{array}{c} {\text{SNRe}}^{\prime }=100*\frac{{\text{SNRe}}_{\text{after}}}{{\text{SNRe}}_{\text{before}}-1},\\ {\text{CNRe}}^{\prime }=100*\frac{{\text{CNRe}}_{\text{after}}}{{\text{CNRe}}_{\text{before}}-1}. \end{array}$$

In the above formula, the larger the SNRe and CNRe values, the higher the image denoising quality, and vice versa. The larger the value of SNRe′ and CNRe′, the faster the image quality growth rate and the more effective the algorithm.

Strain ratio (SR) is one of the indexes to measure the quality of ultrasonic elastic images. SR is the ratio of the axial strain force between the background area and the characteristic area, which reflects the hardness information of the image characteristic area and the background area. When the SR value is small, it means that there is no obvious change in the strain of the image before and after denoising. The specific expression is as follows:

(3) $$\begin{array}{c} \text{SR}=\frac{\Delta \sigma \text{ image }S}{\Delta \sigma \text{ image }U}. \end{array}$$

In the formula, Δ*σ* image *S* represents the axial strain force in the background area of the image, and Δ*σ* image *U* represents the axial strain force in the feature area of the image. *S* and *U* are the same area of the background area and the area intercepted in the feature area.

*(2) Bilateral Filtering*. Bilateral filtering (BF) is a nonlinear filter, and its principle is similar to Gaussian convolution. The difference is that Gaussian filtering only considers the spatial distance relationship in the neighborhood of the two pixels, which makes the processed image blurred and retains the edge information to a certain extent. The bilateral filter takes the spatial distance of the wave and the difference between two grayscale pixels, and the grayscale change of this difference can enhance the edge pixels of the image. Its definition is given by the following formula:

(4) $$\begin{array}{c} BF\left(\mu_{p}\right)=\frac{1}{T_{p}}\sum_{q\in s}H_{\tau_{d}}\left(\left\|p-q\right\|\right)H_{\tau_{r}}\left(\mu_{p}-\mu_{q}\right)\mu_{q}, \end{array}$$

among which

(5) $$\begin{array}{c} T_{p}=\sum_{q\in s}H_{\tau_{d}}\left(\left\|p-q\right\|\right)H_{\tau_{r}}\left(\mu_{p}-\mu_{q}\right). \end{array}$$

*S* is the neighborhood value centered on *p*, and *q* is any pixel in *S*. It is mainly used to measure the amount of denoising of the image; *H*_*τ*_*d*__ is a spatial distance function; *H*_*τ*_*r*__can suppress the influence of pixels far away in space. It is similar in grayscale. The degree function can reduce the influence of different gray values. The definition of*H*_*τ*_*r*__ the neutralization function of *H*_*τ*_*d*__ the bilateral filter is as follows:

(6) $$\begin{array}{c} H_{\tau_{d}}=e^{-\left(1/2\right){\left(d\left(p,q\right)/\tau_{d}\right)}^{2}},\\ H_{\tau_{r}}=e^{-\left(1/2\right){\left(\left(\vartheta \left(I\left(p\right),I\left(q\right)\right)\right)/\tau_{r}\right)}^{2}}. \end{array}$$

In the formula, *d*(*p*, *q*) is the Euclidean distance between the two pixels *p* and *q*, *ϑ*(*I*(*p*), *I*(*q*)) is the grayscale difference between the two pixels *p* and *q*, and *τ*_*d*_ and *τ*_*r*_ are the standard deviation based on the Gaussian function, respectively, and refer to the relative spatial distance and gray value change value of two pixels. In the bilateral filter, the selection of these two parameters has a decisive influence on the denoising performance.

*(3) Heat Conduction Equation*. The partial differential equation processes the image from the perspective of motion. The idea comes from the initial value of the heat conduction equation. The heat conduction equation is as follows:

(7) $$\begin{array}{c} \left\{\begin{array}{c} \partial E\left(m,n,o\right)=\Delta E\left(m,n,o\right),\\ E\left(m,n,0\right)=E_{0}\left(m,n\right). \end{array}\right) \end{array}$$

In the formula, *E*(*m*, *n*, 0) is the original image, and *E*(*x*, *y*, *o*) is the image at time *o* that is being transmitted. The convolution of the Gaussian function and *L*0(*x*, *y*) is the solution of this equation; namely,

(8) $$\begin{array}{c} L\left(m,n,o\right)=G_{\varpi }\left(m,n\right)*L_{0}\left(m,n\right), \end{array}$$

among which

(9) $$\begin{array}{c} G_{\varpi }\left(m,n\right)=\frac{1}{2\pi \varpi^{2}}\exp\left[-\frac{\left(m^{2}+n^{2}\right)}{2\varpi^{2}}\right]. \end{array}$$

In the formula, $\varpi =\sqrt{2t}$. It can be seen from the above formula that the solution of the heat conduction equation at time *t* is Gaussian filtering of the original image; that is, the heat conduction equation at time *t* is equivalent to a Gaussian filter.

(*4) P-M Model*. In order to solve the problem that the heat conduction equation removes noise while also blurring the required edge information, we can naturally think that if the conduction coefficient (i.e., the diffusion coefficient) in the conduction process is adjusted according to the local feature information of the image, it can achieve and automatically identify the edge part of the feature. That is, in the smoother area of the image, the diffusion coefficient can be automatically adjusted to increase, while in the feature edge area of the image, the diffusion coefficient can be automatically adjusted to decrease. In this way, the noise in the smooth area can be effectively suppressed, and the edge information can be better preserved. At the end of the 20th century, Perona and Malik used the gradient as a variable and controlled the diffusion coefficient on the basis of additive noise to obtain a new diffusion model called a nonlinear partial differential equation model (i.e., P-M model). The model is defined as follows:

(10) $$\begin{array}{c} \left\{\begin{array}{c} \frac{\partial E\left(m,n,o\right)}{\partial o}=\text{div}\left(c\left(\left|\nabla E\right|\right)\nabla E\right),\\ E\left(m,n,o\right)=E_{o}\left(m,n\right). \end{array}\right) \end{array}$$

It can be seen from the equation that the larger the value of the spread function, the more smoother the image noise area; when it spreads to the edge of the image and when the spread function value is approximately equal to 0, the edge information of the characteristic area is retained. Perona et al. gave two classic diffusion function definition expressions as follows:

(11) $$\begin{array}{c} \left\{\begin{array}{c} c\left(\left|\nabla E\right|\right)=\exp\left[-{\left(\frac{\left|\nabla E\right|}{k}\right)}^{2}\right],\\ c\left(\left|\nabla E\right|\right)=\frac{1}{\left[1+{\left(\left|\nabla E\right|/k\right)}^{2}\right]}. \end{array}\right) \end{array}$$

In the formula, *k* is the diffusion threshold and ∇*E*can restrain the equation from further diffusion and is the image gradient, which can be used to detect the edge here. If the image gradient value is much larger than the diffusion threshold *k*, the value*c*(|∇*E*|) approaches 0 and the diffusion is suppressed; if the image gradient value is much smaller than the diffusion threshold *k*, the value*c*(|∇*E*|) approaches 1, and the diffusion is enhanced, which is equivalent to a Gaussian filter. Among them, if the selection of the diffusion threshold *k* is too large, excessive smoothing will occur, the image will become blurred, and the edge information of the feature area will be partially smoothed; if the *k* value is selected too small, after several iterations of the denoising model, the smoothing operation stops, which leads to a large amount of noise being retained, and the image denoising effect is not good.

The discrete equation of the P-M model is as follows:

(12) $$\begin{array}{c} Q_{u}^{p+1}=Q_{u}^{p}\lambda \sum_{t\in n}c\left(\left\|Q_{u,t}^{p}\right\|\right)Q_{u,t}^{p}, \end{array}$$

where *Q*_*u*_^*p*^ is the current discrete sampled image, *Q*_*u*_^*p*+1^ is the next discrete sampled image, *u* is the coordinate of the pixel point, *n* is the area with the pixel point *u* as the neighborhood, *t* is any point in the neighborhood, and *λ* is the parameter to control the diffusion. It is usually set to a constant 0.2 in denoising.

Although the PM model is a relatively common denoising method in image processing application research, it still has some shortcomings: spreading at the edge of the image with large changes in grayscale, the smoothing coefficient is too small, and it is easy to cause the edge. The nearby noise points cannot be eliminated; whether the solution of the PM equation exists or is unique, we cannot give an exact answer; the model is unstable; the value of the diffusion threshold *k* is difficult to determine, too large or too small will affect the denoising effect of the image. For the difficult problem of selecting the diffusion threshold *k*, there are usually two solutions: one is to make the *k* value adaptive and automatically obtain the best *k* value. At present, some researchers have achieved corresponding research results in ultrasonic speckle noise reduction; the other is the introduction of parameters; through the introduction of new parameters, the two parameters are mutually restricted to achieve the purpose of noise suppression.

### 2.3. Virtual Reality Technology

#### 2.3.1. Brief Introduction of Virtual Reality Technology

Virtual reality is the sense of virtual reality, referred to as VR for short. Near-field virtual reality technology mainly refers to the data exchange glasses and test gloves equipment between computers and stereo computers and other auxiliary testing devices, so that people can feel the corresponding sense of vision, hearing, touch, intensity, and even smell. This information creates a three-dimensional atmosphere and creates a realistic three-dimensional environment. The general concept of virtual reality has been greatly expanded. It not only includes the above-limited content but also includes all related simulation software and materials, as well as the technology and methods used, for example, “artificial reality,” “virtual environment,” “cyberspace,” and so on. Virtual reality refers to computer graphics, software engineering, medical image processing, image technology, detection and measurement technology, simulation technology, artificial intelligence, pattern recognition, human-machine interface technology, network technology, and real-time distributed processing which can be said to be theoretical technology. It is the product of integration of multiple disciplines.

#### 2.3.2. The Composition of the Virtual Reality System

General virtual reality systems include computer hardware platforms, software systems, input devices, and output devices. People use these devices to obtain information such as sight, hearing, and smell and feel the actual scene.

1. Hardware platform: virtual modeling is a very complex process, so the production of virtual reality scenes has high requirements on the central computer. Due to the real-time requirements of computers, the amount of calculation is very large, and machines with less materials cannot meet the requirements. Currently, foreign virtual reality systems generally have SGI or SUN workstations. Large-scale virtual reality systems use parallel computing systems.
2. Software system: software is the basic technology to realize virtual reality. At present, the representative technologies of VR include X3D, VRML, Java 3D, Cult3D, Viewpoint, Atmosphere and Superscape VRT, EAISense 8 World Tool Kit, and MPI Vega. These are used on the server. The application of virtual reality technology in the virtual medical education system provides tools for its applications.

#### 2.3.3. Main Features of Virtual Reality Technology

The main characteristics of virtual reality technology are immersion, interactivity, and conception. Immersion is also known as presence, which refers to the degree of realism experienced by users in a simulated environment. An excellent virtual reality system must make people feel like they are in a virtual environment, no matter what kind of understanding people have. They need to let people experience real life. This operation performed by the virtual reality system is called “immersion.” This immersion is different from the experience of general computer interactive 3D animation projects. People have a more realistic feeling about wearing stereo eyes and data gloves. Interactivity means that participants can not only passively feel in the virtual environment but also can change or choose emotional content through their own choices. The interactive function of virtual reality can realize the research and function realization of human interaction in the virtual environment. For example, most doctors and students use virtual surgical tools to perform related virtual operations in three-dimensional space. The virtual operating environment generated by the computer can provide operators and salesmen with real-time information and timely intelligence and adjust operations in a short period of time based on feedback. They can repeat the same operation many times or use different strategies for different operations. Conceptuality means that users can imagine the space left by virtual reality technology by themselves. It not only allows participants to have a personal experience but also creates an infinite fantasy space for them. Participants are free to improve their abilities, expand their knowledge, and work boldly. In this way, the virtual reality system provides participants with the ability to actively imagine and create. This conceptual environment of virtual reality is used in the field of education, which can give full play to the enthusiasm of students for inquiry and research.

#### 2.3.4. Application of Virtual Reality Technology in the Medical System

The simulation scene constructed by virtual reality technology can simulate various diseases and different symptoms, which has great research significance and value for the diagnosis and treatment of cardiovascular diseases. Through virtual reality technology, doctors can freely choose pathological conditions and repeatedly train, thereby improving the level of diagnosis and treatment and accumulating clinical experience.  Figure 1 shows the application of virtual reality technology in medicine (this picture is borrowed from Baidu Gallery: https://wenku.baidu.com/view).

## 3. The Clinical Application Experiment of Ultrasound Virtual Reality Technology in the Diagnosis and Treatment of Cardiovascular Diseases

### 3.1. Clinical Experiment Subjects for the Diagnosis and Treatment of Cardiovascular Diseases

This article selects the patients with cardiovascular disease received from Y Hospital in China from April 2018 to April 2019 as the research object, with a total of 86 patients. The experimental subjects were divided into experimental group and control group, with 50 cases and 36 cases, respectively.

### 3.2. Inclusion Criteria

1. All meet the relevant standards and classification schemes of cardiovascular diseases, have clear consciousness, and are 20–80 years old
2. They are admitted to the hospital for treatment because of being diagnosed as a cardiovascular disease
3. All experiments were carried out with the informed and consent of the patients

According to the order of admission, they were randomly divided into two groups: the control group was treated with traditional medicine, and the observation group was treated with ultrasound virtual reality technology. The two groups had no statistically significant differences in age, gender, medical history, course of disease, etc. (*P* > 0.05), and they were comparable.  Table 1 shows the basic pathological data of the patients.

### 3.3. Exclusion Criteria

1. The patient is a pregnant woman
2. A history of allergy to cardiovascular ultrasound diagnosis
3. Impairment of liver and kidney function
4. Suffering from mental illness and other diseases
5. The age being less than 20 years or more than 80 years

### 3.4. Treatment Methods

For the treatment of all patients with cardiovascular diseases, the main equipment is GE730. The probe frequency is 3∼5 Hz. The patient is placed on his back and lying on the examination table. The ultrasound Doppler is used for the examination. The examination time is longer and the patient needs to be told. Let the patient fully expose the affected side, check carefully from top to bottom, to avoid omissions, mainly scan the bilateral common arteries, branch veins, and arteries, pay attention to whether there are emboli, use images to record, and make the blood vessels shape and wall thickness to record.

### 3.5. Observation Indicators

The main observation indicators studied in this paper are the detection, missed detection, and misdiagnosis of the patient's disease using ultrasound virtual reality technology before treatment, the recovery of various physical indicators of the patient after treatment, and the adverse reactions after the operation.

### 3.6. Statistical Methods

The statistical method uses SPSS22.0 statistical software, the measurement data are expressed as mean ± standard deviation (*x* ± *s*), the comparison of measurement data between groups uses *t*-test, the comparison before and after itself uses paired *t*-test, and the count data use chi-square test. *P* < 0.05 indicates that the difference is statistically significant.

## 4. The Clinical Application of Ultrasound Virtual Reality Technology in the Diagnosis and Treatment of Cardiovascular Diseases

### 4.1. Application Field Analysis of Virtual Reality Technology

In the context of the continuous development of the virtual reality industry, the virtual reality industry has been involved in various fields and has played a greater role. The practical activities in virtual reality provide humans with a wider range of applications. Nowadays, virtual reality can be seen to shine in all aspects of production and life. As can be seen in Table 2 and Figure 2, the estimated revenue and application proportions of VR technology in different application fields, it can be seen that the current virtual reality technology has been used in entertainment, military, industry, education, real estate, retail, health care, live broadcast, etc. All fields are involved. Among them, the highest proportion of revenue is in the entertainment field. Virtual reality technology can transform all two-dimensional images, pictures, and games into three-dimensional scenes, which can be interacted with in real time. This meets the needs of humans for high-level human-computer interaction and also allows users to fully enjoy the immersion in entertainment The happiness of the world. At present, VR movies, VR tourism, VR live broadcast, VR concerts, and VR games are all adding vitality to human entertainment life, and more and more entertainment projects are moving towards the “+VR” ranks.

### 4.2. Technical Comparison and Analysis of Ultrasonic Virtual Reality

It can be seen from Table 3 and Figure 3 that the cost-sensitive feature sampling algorithm has less sampling cost than random sampling (different sampling ratio), and the advantage is more obvious when the proportion of missing attribute values is higher. When the attribute missing rate is 20%, the cost of the cost-sensitive feature sampling algorithm in this chapter is only slightly less than the cost of 25% random sampling, but when the attribute value missing reaches 80% and 100%, the cost of the algorithm in this chapter is much less than random sampling. And when the sampling cost is taken into consideration, it can be seen that the comprehensive cost of random sampling increases as the sampling ratio increases, and the difference between them increases rapidly with the increase in the proportion of attribute missing. This shows that random sampling does not bring significant performance improvement when there is more redundancy for attributes such as hypertension, and the overall classification cost performance deteriorates due to the increase in sampling cost. However, the cost-sensitive active learning method in this chapter can first discover and sample the attributes related to the classification task. On the one hand, it reduces the number of samples. On the other hand, the high quality of the sample improves the classification accuracy. It also brings a reduction in the cost of classification errors. Experiments show that the algorithm in this chapter has achieved a good balance between the attribute sampling cost and the misclassification cost, making sampling cost + misclassification cost significantly reduced compared to random sampling.

It can be seen from Table 4 and Figure 4 that, from subjective vision, we can clearly see that the algorithm in this paper performs more prominently in terms of noise smoothing ability when the edge information of the feature area is kept approximately the same. It can also be seen from the SNRe and CNRe curve changes that the SNRe and CNRe values of the ultrasonic elastic images after filtering have been greatly improved, and when the number of iterations is 100, SNRe and CNRe tend to be stable values.

### 4.3. Experimental Results

It can be seen from the data acquisition in Table 5 and Figure 5 that the incidence of hypertension and related risk factors in hypertensive patients were investigated using the multidimensional random sampling method. Basic information includes pathological status, family genetics, action risk factors, health awareness about high blood pressure, and measurement of height, weight, waist circumference, blood pressure, etc. The survey results showed that the total prevalence of hypertension was 25.1%, 25.9%, and 24.4% for men and women and 32.0%, 21.5%, and 23.6% for rural, urban, and urban areas.

As can be seen from Table 6 and Figure 6, the experimental group uses ultrasound virtual reality technology for diagnosis, and the control group uses traditional diagnostic methods. From the survey data, 42 cases were detected in the experimental group, reaching a diagnosis accuracy rate of 85.39%, while the number of detection in the control group was 24 cases, which was 76.8%. In addition, in terms of the missed detection rate and the misdiagnosed rate, the control group has more than 20%, while the experimental group does not exceed 5%. This shows that the use of ultrasound virtual reality technology for disease diagnosis can improve the diagnostic accuracy of cardiovascular diseases and reduce the proportion of misdiagnosis and missed detection.

It can be seen from Figure 7 and Table 7 that the clinical manifestations of cardiovascular disease include heart palpitations, chest pain, headache, vomiting, and paralysis. The experimental group and the control group have significant improvements before and after treatment, but the experimental group's treatment effect is far higher than the control group. Take heart palpitations as an example. Before treatment, the symptoms of the experimental group reached 90.1%, and the proportion of the control group before treatment was 97.6%; after treatment, the palpitations of the experimental group dropped to 47.6%, while the control group still had 70.1% of patients having this kind of performance, so, in comparison, the treatment effect of the experimental group is better than that of the control group.

As shown in Table 8 and Figure 8, the postoperative state of the two groups was compared. Patients in both groups underwent VAS pain scores after surgery. The average score of the experimental group was lower than that of the control group (*P* < 0.05). The incidence of complications during and after the use of antibiotics was significantly lower than that of the control group (*P* < 0.05). After a year of follow-up investigation, the recurrence rate of the experimental group was lower than that of the control group, and the difference was statistically significant (*P* < 0.05).

## 5. Conclusion

This article mainly studies the clinical application of ultrasound virtual reality technology in the diagnosis and treatment of cardiovascular diseases. Through an in-depth understanding of virtual reality technology, we determine the feasibility and necessity of virtual reality technology in the diagnosis and treatment of cardiovascular diseases. For the medical industry, it is a research in a new direction, which has certain significance and practical value.

This article mainly uses the literature method, experimental analysis method, and other methods to discuss and apply ultrasonic image denoising algorithm and design the application experiment of cardiovascular disease diagnosis and treatment based on ultrasonic virtual reality technology. The main innovations of this article are the combination of theory and practice, the full application of theoretical foundations in practice, and the application of virtual reality technology to the diagnosis and treatment of cardiovascular diseases; second, the combination of qualitative and quantitative research is used, with both data analysis and qualitative content analysis.

This article still has some shortcomings, such as the experimental period is not long enough and the experimental subjects are not wide enough. The research data still need to be improved and viewed more comprehensively. The research in this article is an innovation for medicine and VR technology. In the future, as the development of VR technology becomes more and more mature, it will also promote the development of more industries.

## Figures and Tables

**Figure 1:** Application of virtual reality technology in medicine.

**Figure 2:** The proportion of applications of virtual reality technology in various fields.

**Figure 3:** Comparison of the cost of feature collection for hypertension data with different attribute missing proportions.

**Figure 4:** SNRe and CNRe values before and after ultrasound image filtering.

**Figure 5:** The average value and standard deviation of some important indicators in the hypertension survey data of the surveyed patients.

**Figure 6:** The diagnostic accuracy rate of ultrasound virtual reality technology for cardiovascular diseases.

**Figure 7:** Comparison of clinical manifestations between the experimental group and the control group before and after treatment (%).

**Figure 8:** Comparison of postoperative conditions between the two groups.

**Table 1:** Comparison of patient pathology data.

Basic information	Control group	Test group
Male	20	25
Female	16	25
Age < 45	6	6
45–65	12	20
Age > 65	4	12
Medical history 1–3 years	26	22
Medical history more than 3 years	10	28

**Table 2:** The proportion of applications of virtual reality technology in various fields.

Field classification	Proportion of application usage	Revenue as a percentage
Military	10.09	3.28
Engineering	12.01	4.75
Medical treatment	7.61	5.18
Education	9.32	0.79
Real estate	12.58	2.69
Retail	3.43	1.67
Live broadcast	11.31	4.11
Entertainment	37.92	3.26

**Table 3:** Comparison of the cost of feature collection for the hypertension data with different attribute missing proportions.

Proportion of missing attribute values (%)	20	40	60	80	100
Random sampling (25%)	203	219	498	611	980
Random sampling (50%)	159	437	772	1229	1684
Random sampling (75%)	384	526	1232	1668	2689
Cost-sensitive sampling	134	158	198	222	234

**Table 4:** SNRe and CNRe values before and after ultrasound image filtering.

Method	Window size	Number of iterations	SNRe	CNRe	Up SNRe	Up CNRe
Image A	—	—	6.564	3.413	—	—
Image B	3 × 3	100	21.364	10.378	225.411	213.741
Image C	3 × 3	100	23.415	11.681	256.624	243.232
Image D	5 × 5	100	26.833	13.234	308.693	288.875
Image E	—	—	9.623	6.813	—	—
Image F	3 × 3	100	16.728	13.098	94.112	92.265
Image G	3 × 3	100	17.012	13.324	97.413	95.532
Image H	5 × 5	100	17.017	13.318	98.565	95.345

**Table 5:** The average value and standard deviation of some important indicators in the hypertension survey data of the surveyed patients.

Index	Mathematical expectation	Variance	Covariance	Standard deviation
Age	41.43	1.93	2.22	2.01
Gender	1.53	2.15	1.88	2.02
Smokes	1.63	1.92	2.21	2.05
Annual family income	3.66	1.82	2.01	2.43
Excessive alcohol intake	1.69	2.16	2.48	1.81
BMI	22.14	2.29	1.93	2.48
Family history of hypertension	1.13	1.8	1.98	2.34
Lack of physical exercise	1.98	2.47	2.32	2.31
Marital status	1.34	2.35	2.14	2.06
Education level	2.36	3.14	2.39	2.01

**Table 6:** The diagnostic accuracy rate of ultrasound virtual reality technology for cardiovascular diseases.

Grouping	Number of people checked out	Detection ratio	Number of misdiagnosed	Misdiagnosis ratio	Number of missed inspections	Proportion of missed inspections
Test group	42	85.39	3	1.76	5	2.23
Control group	24	76.8	4	9.85	8	13.28
*T* value	3.48	2.76	2.83	3.45	2.87	2.77
*P* value	3.22	3.3	3.33	3.29	3.4	3.71

**Table 7:** Comparison of clinical manifestations between the experimental group and the control group before and after treatment (%).

Index	Test group		Control group	
	Before therapy	After treatment	Before therapy	After treatment
Heart palpitations	90.1	47.6	97.6	70.1
Chest pain	72.6	22.6	75.0	38.5
Headache	55.1	22.6	67.6	25.1
Vomiting	47.6	20.1	45.2	35.1
Hemiplegia	55.8	10.9	46.9	33.2
Shortness of breath	68.9	33.2	69.7	45.1

**Table 8:** Comparison of postoperative conditions between the two groups.

Group	Number of cases	Postoperative pain score (VAS)	Postoperative exhaust time (d)	Antibiotic use time (d)	Incidence of postoperative complications (*n* (%))	The recurrence rate was followed up for 1 year (*n* (%))
Test group	50	2.8	1.7	2.1	1 (4.76)	2 (9.52)
Control group	36	3.7	2.1	3.2	7 (33.33)	9 (42.86)
*T* value	—	2.2367	2.1309	2.6830	—	—
*X*2 value	—	—	—	—	3.8603	6.0353
*P* value	—	<0.05	<0.05	<0.05	<0.05	<0.05

## Data Availability

No data were used to support this study.
